# The Impact of Headgear on Distalization in Class II Division I Malocclusion: A Case Report

**DOI:** 10.7759/cureus.52213

**Published:** 2024-01-13

**Authors:** Samer Mereani, Reaam K Indijani, Amjad Alotaibi

**Affiliations:** 1 Orthodontics, King Faisal Hospital, Mecca, SAU; 2 General Dentistry, King Abdulaziz University, Jeddah, SAU; 3 General Dentistry, King Abdulaziz Medical City, Ministry of National Guard Health Affairs, Jeddah, SAU

**Keywords:** orthodontics, headgear, distalization, appliance, expansion

## Abstract

This report presents a case of a 16-year-old female patient with skeletal class II and dental class II division I malocclusion that was treated with fixed orthodontic appliances and through growth modulation. Two appliances were used: a Hyrax expander and a high-pull headgear with extraction. The treatment objectives of achieving a class I molar and canine relationship, resolving the crowding in the upper and lower arches, correcting the midline shift, and improving the patient's facial profile and lip position were achieved, resulting in a good occlusion with normal overbite and overjet.

## Introduction

Class II malocclusion is one of the most commonly encountered problems in orthodontic practice. It is associated with functional, esthetic, and psychological issues of varying intensities [1]. Skeletal class II malocclusions are among the most prevalent malocclusions and can involve maxillary protrusion, mandibular retrusion, or a combination of both. However, mandibular retrusion is a major contributory factor in around one-third of skeletal class II malocclusion cases [2]. Moreover, skeletal class II malocclusion can conceal a transverse maxillary deficiency, which is typically treated with rapid palatal expansion (RPE) [3]. The most effective method for treating skeletal-based conditions in adult patients is a combined orthognathic-orthodontic approach. However, surgery may not be feasible for many of these patients due to medical or financial concerns [4]. In such cases, alternative options should be considered. Various functional appliances have been used in the management of class II malocclusion [5]. For instance, headgear has been used for a long time and has a range of therapeutic applications in modern orthodontics, such as molar distalization, maxillary growth restriction, and anchoring management. The force applied by a headgear for molar distalization should be consistent and stable to allow for effective tooth movement. It should be relatively light as it primarily targets the first molars. The recommended force is around 100 grams, enabling a tooth movement rate of 1 mm per month. The duration of wear should be as long as possible, as wearing the device more frequently leads to better and faster results. The minimum recommended period for wearing headgear is 14 to 16 hours per day [6-7]. When the maxilla moves, the force vector should pass through the center of resistance of the maxilla to achieve bodily movement. A high-pull headgear can be used to minimize the forward and downward movements of the upper molars [5].

## Case presentation

A 16-year-old female presented to the Department of Orthodontics at King Faisal Hospital, mecca, Kingdom of Saudia Arabia, with a primary concern of her upper front teeth protruding. She exhibited a convex facial profile and a mandibular deficiency. Her smile appeared fairly symmetrical, but she had a non-consonant smile arc and excessive display of maxillary gingiva when smiling (Figure 1).

**Figure 1:** Pre-treatment extraoral and intra-oral photographs (A) Incompetent lips. (B) Inconsonant smile arch. (C) Facial profile: right lateral view showing the NLA line tangent to the base of the nose and a line tangent to the upper lip (red arrow); E-line is drawn from Pn (point of the nose) to pog (soft tissue pogonion) (black arrow). (D) Increased overjet. (E) Frontal view showing diastema. (F) Left lateral view showing increased overjet. (G, H) Occlusal view showing crowding in the upper and lower arches. NLA, nasolabial angle

Cephalometric analysis revealed skeletal anteroposterior dysplasia due to mandibular deficiency (ANB: 7.0°), characterized by a steep mandibular plane angle and slightly increased lower facial height (ANB = SNA-SNB, where SNA is sella, nasal, anterior of the maxilla and SNB is mean mandible. This angle relates the anterior limit of the maxillary bone [point A] and mandibular bone [point B] with the anterior limit of the nasofrontal suture [point N]. The ANB angle measures the relative anteroposterior position between the maxilla and mandible). The maxillary incisors were positioned anteriorly in relation to the A-pogonion line (Table 1). The patient exhibited normal positioning of the upper and lower lips in relation to the E-line, with an acute nasolabial angle (NLA). Intra-oral examination and study casts indicated a bilateral class II molar and canine relationship, along with a posterior cross-bite. The lower dental midline was shifted 5 mm to the right in relation to the facial midline, while the upper dental midline was aligned. The patient had proclined upper incisors with an overjet of 10 mm. In addition, there was an impacted lower right second premolar and congenitally missing upper first premolars. The upper and lower arches exhibited dental crowding of 1 mm and 8 mm, respectively. The final diagnosis was skeletal class II division I malocclusion with transverse maxillary deficiency (Figures 2-4).

**Table 1:** Post-treatment lateral cephalometric analysis ANB, anteroposterior position between the maxilla and mandible; Inc, incisor; L, lower; Mand, mandibular; NA nasion (point A); NA-APg, nasion (point A) and pogonion; NB, nasion to point B; NPg-FH, nasion to pogonion on Frankfort horizontal plane; Occ, occlusal; SN, sella nasion line; SNA, sella and nasion (point A); SNB, sella and nasion (point B); U, upper

Area of study	Measurement	Mean	Pre-treatment	Progress	Post-treatment
Sagittal relationship	NPg.-FH	87° ± 3	85°	86°	86°
	SNA	82° ± 3 °	77°	78°	78°
	SNB	80° ± 2	70°	72°	73°
	ANB	02° ± 2	7°	6°	6°
	NA-APg.	01° ± 04	9°	6°	6°
	*Wits appraisal	0 mm	6mm	5mm	4mm
Vertical relationship	Mand. plane to FH	22° ± 5	29°	30°	31°
	Mand. plane to Sn	32° ± 5	38°	39°	40°
	Occ. plane Sn	14° ± 5	22°	23°	23°
	Lower face height	55% ± 2	57%	58%	58%
Dental relationship (incisor position)	U Inc. to Sn	103° ± 7	114°	112°	108°
	U Inc. to NA	22° ± 6	29°	28°	26°
	U Inc. to NA (mm)	6 mm ± 2	9mm	8 mm	6mm
	U Inc. to L Inc.	130° ± 9	118°	119°	123°
	L Inc. to Mand.	93° ± 6	93°	93°	95°
	L Inc. to NB	25° ± 6	29°	31°	33°
	L Inc. to NB (mm)	4 mm ± 2	5mm	6mm	7mm
	L Inc. to APg. (mm)	1 mm ± 2	2mm	3mm	4mm
Soft tissue relationship	U lip to E-line	-4 mm ± 2	-1 mm	-4 mm	-5 mm
	L lip to E-line	-2 mm ± 2	+1 mm	0mm	-1 mm
	Nasiolabial angle	90-110°	87°	84°	88°

**Figure 2:** Pretreatment dental cast

**Figure 3:** Pretreatment lateral cephalometric and panoramic radiographs

**Figure 4:** Lateral cephalometric radiographs showing the mandibular angle, pogonion line, and lower facial height (A) Lower facial height: The ratio of the distances G-Sn and Sn-Me; in normal cases, it should be approximately 1:1. (B) Frankfort-mandibular plane angle (FMA) is formed by the intersection of the Frankfort horizontal plane (FH plane) and the mandibular plane (1). Pogonion line is a line to measure the position of the anterior teeth (2). G-Sn, glabella to subnasale; Sn-Me, subnasale to menton

Treatment objectives

The treatment objectives were as follows: (i) to achieve a bilateral class I molar and canine relationship by performing extraction and using high-pull headgear and fixed appliance, (ii) to reduce anteroposterior skeletal discrepancy and improve the facial profile by obtaining an ideal overjet and aligning the teeth, (iii) to reposition the lower right lateral, a transposition tooth, to its normal position, and (iv) to use a Hyrax expander for plate expansion and correction of posterior crossbites.

Treatment alternatives

Orthognathic surgery was initially considered as the primary treatment option. However, the case was ultimately managed using a comprehensive orthodontic treatment plan, which included fixed appliances, in accordance with the parent’s preference. Additionally, high-pull headgear, rapid palatal expander, and teeth extraction were incorporated into the treatment approach. Although temporary anchorage devices was the best option in this case, it was not available as an option during the treatment of this case.

Treatment progress

Pre-treatment data were collected, and diagnostic records were analyzed before the treatment. The patient and her guardians were informed about the importance of maintaining good dental hygiene, as well as the benefits and risks associated with this treatment method.

As the patient had skeletal class II malocclusion, the treatment was initiated with the implementation of a palatal expansion appliance (Hyrax expander) to create space for the congenitally missing teeth (#14 and #24), improve the upper arch shape, and correct posterior crossbites. The Hyrax expander was cemented and activated once daily for the first five days. Subsequently, it was continuously activated with two turns per day for four months. Following this period, the appliance was used as a stabilizer for an additional four months.

After removing the Hyrax expander, a high-pull headgear was used to move the upper molars distally and restrict the growth of the maxilla. The headgear exerted a force of 200 g per side for the first month and 400 g thereafter. It was recommended to wear the headgear for 12 to 14 hours daily. After eight months of headgear use, space was created in the maxillary arch (2 mm/side) to attach two segmented archwires ON the right and left sides including canines and premolars with 0.012 nickel-titanium (NiTi) archwire, while 0.012 NiTi archwire was placed for the lower teeth. The headgear was removed after 14 months, and preadjusted, edgewise, fixed appliances with MBT (MacLaughlin, Bennet, and Trevisi) brackets (3 M Gemini MBT 0:022′′ × 0:028′′ slot size) were placed on the lower and upper teeth with 0.014 NiTi archwire. The headgear was still used at night for anchorage (Figures 5, 6).

**Figure 5:** Treatment progress (A) Picture showing insertion of the high-pull headgear. (B) Image after the end of expansion. (C) Occlusal photograph showing the hyrax expander.

**Figure 6:** After one year and two months of wearing headgear Represent lateral view (A, B). Lower occlusal view shows the lower segmented arch with 0.014 NiTi (C) and the upper segmented arch with 0.018 NiTi (D). NiTi, nickel-titanium

To create space for the blocked lateral incisor and correct the 5-mm midline shift to the right in the mandible arch, the left first premolar was extracted, and the archwire was changed to 0.019 × 0.025 stainless steel (SS) wire with a push coil between the right central incisor and the right canine. On the opposite side, a power chain was placed from the left canine to the left first molar, along with a class III elastic (1/4 in diameter, 2 oz), to address the anteroposterior discrepancy and establish the mandibular arch length. Once sufficient space was achieved, the right lateral incisor was brought into the arch by bonding a button lingually and using a power chain from the mandibular right central incisor to the mandibular right canine, passing through the button of the lateral on a 0.018 SS archwire. During this phase, a power chain was used from the maxillary right canine to the left canine in an attempt to close the diastema (Figure 7).

**Figure 7:** Intra-oral view after creating space in the lower teeth (A) Upper occlusal 0.019 x 0.025 SS archwire with powerchain from 3-3 (upper right canine to upper left canine). (B, C) After create space for the lateral start bring it to the arch (bond button lingually to the lower right lateral and powerchain from lower first central to canine and pass through the button of lateral on 0.018 SS arch wire. SS, stainless steel

In the final phase of treatment, both the upper and lower arches had a 0.019 × 0.025 SS wire with torque added to the lower right lateral incisor. In the maxillary arch, steel colligation was placed from the right first molar to the left first molar. Kobayashi ligatures were also added to both the right and left laterals to hold elastics in place. Specifically, zigzag elastics with class II components on both the right and left sides (5/16 in diameter, 2.5 oz) (Figure 8) were used to correct the anteroposterior relationship of the dentition and to improve interdigitation, resulting in a more stable occlusal correction.

**Figure 8:** Final phase of the treatment A, B) Adding Kobayashi ligature to upper right and left lateral view for elastic holding zigzag elastic with class II component right and left (5/16 in diameter, 2.5 oz). (C, D) Both the upper and lower arches had 0.019 x 0.025 SS with steel colligation from 6-6 (from the upper right first molar to the upper left first molar).

The following factors were taken into account when considering this potential treatment option. Because of the maxillary teeth crowding and posterior crossbites caused by the high, arched, V-shaped palate, a rapid palatal expander and high-pull headgear were used initially. As a result, a 5-mm space was created on each side as the palate expanded, and the molar distalization effectively addressed the crowding and reduced the overjet. In addition, a comprehensive extraction orthodontic treatment was employed to correct the midline shift and resolve severe crowding (8 mm) by bringing the blocked lower right lateral into the arch.

After 36 months of active treatment, the fixed appliances on the maxillary and mandibular were removed, and post-treatment records, such as cephalometric X-rays (Orthophos XG, Mecca, Saudi Arabia), panoramic radiographs (Orthophos XG), impressions, and photographs (Canon Mark II with a 90-mm macro lens), were acquired to assess the success of the treatment objectives. We opted for a fixed retainer in the form of upper and lower wraparound retainers, extending from canine to canine, due to the presence of diastema and crowding in the upper and lower teeth.

Improvements in the patient’s facial profile and lip position were observed. The post-treatment facial photographs showed a significant change in the upper lip posture in relation to the E-line, indicating that it has become competent (Figure 9). Intra-oral findings and the post-treatment casts revealed well-aligned arches and proper interdigitation of the dentition. In addition, class I canine and class I molar relationships were maintained with good overjet and overbite. All maxillary spaces, including the diastema, were closed, and lower crowding was corrected. The lower right lateral incisor was successfully aligned into the arch. The upper and lower dental midlines coincided with the facial midline (Figure 9).

**Figure 9:** Post-treatment extra-oral and intra-oral photographs (A) Lips position improved and became competent. (B) Consonant smile arch. (C) Improved facial profile and NLA. (D) Right lateral view showing the achieved minimum overjet. (E) Frontal view showing improved midline shift and close diastema. (F) Left lateral view showing the achieved minimum overjet. (G, H) Occlusal view results in resolved crowding in the upper and lower arches. NLA, nasolabial angle

From a periodontal point of view, the case showed generalized gingivitis with mucogingival deformity. After orthodontic treatment, the conditions of the oral mucosa and gingiva improved significantly, and the disease was effectively managed. The patient achieved appropriate occlusion and a healthy oral environment. Nevertheless, it is still necessary for the patient to visit the periodontal clinic to address gingival recession at teeth #13, #23, and #43.

An end-treatment panoramic radiograph indicated that all roots were well-aligned, except for the lower right canine (Figure 10).

**Figure 10:** Final panoramic view

A post-treatment cephalometric evaluation and superimposed cephalometric tracing revealed a decrease of 2° in the ANB angle, but the skeletal relationship remained to be class II. Moreover, an acceptable NLA was achieved as the upper incisors retruded and retroclined by about 5°, while the lower incisors proclined. The mandibular plane angle and the lower facial height slightly increased due to mandible growth and autorotation (Table 1). During the three-year retention follow-up, the patient’s occlusion and facial esthetics were stable (Figures 11, 12).

**Figure 11:** Initial and final lateral cephalometric radiographs

**Figure 12:** Superimposition of the maxilla and mandible The black line indicates pre-treatment, and the red line indicates post-treatment 1, molar; 2, incisor; 3, pogonion; 4, gonion

Overall, the treatment was considered successful, and the patient expressed satisfaction with the results.

## Discussion

RPE has been used for over a century as a treatment for maxillary constriction [7]. In this case, a Hyrax expander was initially used to address the patient’s maxillary transverse deficiency and teeth crowding without the need for extraction. By widening the upper dental arch, we increased the intermolar width and arch length, corrected the axial inclination of the posterior teeth, and improved the patient’s smile. Specifically, the maxillary intermolar width increased from 28 mm (pre-treatment) to 35 mm (post-treatment). While RPE created more space, additional space was needed to correct the class II division I dental relationship. The use of high-pull headgear with a fixed appliance is a common treatment plan for growing individuals with class II malocclusion. The orthopedic goal of headgear treatment is to correct dental malocclusion, normalize anteroposterior skeletal relationships, and improve or prevent the worsening of vertical skeletal relationships [8]. A recent study confirmed that the inclination of the palatal plane and the sagittal position of the maxilla remained stable during the post-treatment period, with favorable mandibular development in both the sagittal and vertical planes facilitating class II correction and retention [9]. In this case report, the high-pull headgear moved the upper molar teeth backward by 2 mm on each side and restrained maxillary growth. Therefore, the space gained from functional appliances helped reduce the overjet, address crowding, and correct the class II relationship. The results demonstrated positive changes in both dental and skeletal aspects. The upper incisors were moved backward, resulting in a decrease of 2° in the ANB angle, although it still indicated a class II skeletal relationship. The NLA improved as the upper lip moved backward and the tip of the nose moved forward and downward. A more balanced facial appearance and improved lip competence were achieved at the end of the treatment. The increase in the mandibular plane angle and lower facial height indicated mandibular growth and auto-rotation. Satisfactory functional and esthetic outcomes were achieved without significant injuries. The upper and lower teeth were leveled and aligned without compromising soft tissue and periodontal structure.

Our therapeutic approach has certain limitations, such as a lengthy treatment period and the need for the patient's cooperation in wearing functional appliances. Despite the absence of significant gingival recession, we committed to moving the teeth as slowly as possible in an attempt to prevent rapid tipping of the teeth and minimize the risk of bone dehiscence and root resorption. The results showed no significant gingival recession or major problems. However, the patient was advised to seek treatment for the initial gingival recession.

## Conclusions

The results of this case report demonstrate that class II division I malocclusion can be treated using a high-pull headgear with a fixed appliance and through growth modulation. This approach also improves the soft tissue profile and enhances lip competence. It is crucial to carefully select cases as the application of knowledge, skills, and good patient cooperation ensures a stable, long-term outcome.
